The article "Status of Iodized Salt Coverage in Urban Slums of Cuttack City, Orissa" was published in 2009. Journal: Indian J Community Med.

# Status of Iodized Salt Coverage in Urban Slums of Cuttack City, Orissa

**DOI:** 10.4103/0970-0218.51228

**Published:** 2009-04

**Authors:** Ansuman Panigrahi, Kaushik Mishra, Bijayeeni Mohapatra

**Affiliations:** Department of Community Medicine, Kalinga Institute of Medical Sciences, Bhubaneswar, India; 1 Department of Community Medicine, S.C.B. Medical College, Cuttack, India

**Keywords:** Iodized salt, mental retardation, sustainable elimination, urban slum

## Abstract

**Background:**

For sustainable elimination of iodine deficiency disorders (IDD), it is necessary to consume adequately iodized salt on a regular basis and optimal iodine nutrition can be achieved through universal salt iodization.

**Objective:**

To assess the extent of use of adequately iodized salt in the urban slums of Cuttack.

**Materials and Methods:**

Using a stratified random multi-stage cluster sampling design, a cross-sectional study involving 336 households and 33 retail shops selected randomly from 11 slums of Cuttack was conducted in 2005. A predesigned pretested schedule was used to obtain relevant information and salt iodine was estimated qualitatively by using a spot testing kit and quantitatively using the iodometric titration method.

**Statistical Analysis:**

Proportion, Chi-square test.

**Results:**

Only 60.1% of the households in urban slums of Cuttack were using adequately iodized salt i.e., the iodine level in the salt was ≥15 ppm. Iodine deficiency was significantly marked in sample salts collected from katcha houses as compared with salts collected from pucca houses. Households with low financial status were using noniodized/inadequately-iodized salt. Both crystalline and refined salts were sold at all retail shops. Crystalline salts collected from all retailers had an iodine content < 15 ppm and refined salts collected from one retailer had iodine content < 15 ppm. About 48.5% of salt samples collected from retail shops were adequately iodized.

**Conclusion:**

In the urban slums of Cuttack, retailers were selling crystalline salts, which were inadequately iodized- this would be a setback in the progress towards eliminating IDD.

## Introduction

Iodine deficiency is the world's single most significant cause of preventable brain damage and mental retardation. The clinical and sub clinical manifestations of iodine deficiency are collectively included in the term iodine deficiency disorders (IDD) and affect all stages of human growth and development.(1–3) It also reduces productivity in livestock.(1–3) Thus, to ensure the elimination of iodine deficiency disorders, the national iodine deficiency disorder control program was launched in 1992 with an aim toward universal salt iodization (USI) so that every human would consume adequately iodized salt on a daily basis from now on.(1,4)

About 2.5 lakh tons of salt is imported annually from outside Orissa (mainly Gujrat, Rajastan, Tamil Nadu, and Andhra Pradesh) whereas 0.5 lakh tons is produced inside the state mainly in three districts i.e., Ganjam, Balasore, and Puri. There are eight iodization plants in Orissa (7 in Ganjam and 1 in Balasore). In Cuttack, approximately 35 racks i.e., 84,000 tons of salt are unloaded every year, out of which 10 racks i.e., 24,000 tons contain refined salt.

The urban slum population is such a neglected, underserved section of the society that they are constantly being deprived of various privileges. They live in unhygienic environmental conditions and are always at risk for various health hazards. Lower socio-economic status, lower literacy rate, poverty, ignorance, and a continuous trauma of neglect perpetuate the problems of under nutrition of which iodine deficiency is one of the major nutritional problems. Keeping the above facts in view, this study was conducted to assess the extent of use of adequately iodized salt in the urban slums of Cuttack.

## Materials and Methods

This study was conducted in the urban slums of Cuttack between 1 August 2005 and 31 December 2005 using a stratified random multi-stage cluster sampling design. The sample size of 285 was estimated using the proportion of households utilizing adequately iodized salt as 45% at 95% confidence interval with 10% absolute precision and design effect 3.

Cuttack was divided into 4 geographical divisions i.e., North West, South West, North East, and South East. Each division consists of wards with or without slum areas. Thus, of the wards with slum areas in each division, 25% of the wards were selected using a simple random sampling technique. From each selected ward, one slum area was chosen randomly and in each selected slum area, 10% of the households were selected using a simple random sampling technique. All the selected households were visited by the investigator and relevant information was collected using the predesigned and pretested schedule. Cooperative, willing adult women in the family were approached and information on housing pattern, environmental conditions, type of salt used, and the practice of storing it were collected. Salt samples of approximately 15 grams were collected in sealed polythenes from 336 selected households. To obtain additional information regarding the availability of iodized salt in slum areas, 3 retail shops from each slum area were selected randomly and 2 salt samples each of approximately 15 grams were collected from every retail shop. The retailers were interviewed to determine the type of salt sold, the type of packing used, and the practice of storing salt. The iodine content of salt was determined qualitatively using a spot testing kit to show the study respondents/retailers on the spot whether the salt consumed/sold by them was iodized and also quantitatively by the titration method to assess the extent of use of adequately iodized salt.

## Results

Out of 336 houses, 252 (75%) were katcha houses and 84 (25%) were pucca houses. Of the 336 households, only 186 (55.4%) were using refined (branded, packeted) salt, 130 (38.7%) were using crystalline (loose) salt, and 20 (5.9%) were using powdered (loose) salt. In a majority (82.7%) of the households, salt was stored in containers with lids whereas 17.3% of the households were storing salt in containers without lids.

The iodine content in salts used in the households was determined using the iodometric titration method. From among 336 households, 80 (23.8%) were using noniodized salt and 54 (16.1%) were using inadequately iodized salt; whereas 202 (60.1%) households were using adequately iodized salt i.e., the iodine level in the salt was ≥ 15 ppm [Table 1].

**Table 1:** lodometric titration of sample salt at household level

lodometric titration	Number	Percentage
0 ppm	80	23.8
<7ppm	50	14.9
7–1 4.99 ppm	4	1.2
15–29.99ppm	44	13.1
≥ 30 ppm	158	47.0
Total	336	100.0

Table 2 shows the association of house type, income, and storage practice with the iodine content of sample salts collected from households. It was observed that the iodine deficiency in sample salts was predominantly marked in the katcha houses i.e., 120 (47.6%) as compared with pucca houses i.e., 14 (16.7%) and this difference was found to be statistically significant. Again, the iodine deficiency in the sample salts was marked more in households with low per capita monthly income i.e., 120 (47.3%) as compared with those in the middle-income group i.e., 14 (17.1%). The iodine content was ≥15 ppm in 190 (68.4%) sample salts stored in containers with lids as compared with 12 (20.7%) sample salts stored in containers without lids. The iodine level was < 15 ppm in 46 (79.3%) sample salts stored in containers without lids as compared with 88 (31.6%) samples that were stored in containers with lids. This difference was found to be statistically significant.

**Table 2:** Type of house, per capita monthly income, storage practice and salt iodine level

		Iodine content in salt (in ppm)	Chi square value	*P* value
			
	<15	≥15		
House type				
Pucca	14	70		
Kutcha	120	132		
Total	134	202	12.58	*P*<0.001
Income								
Low	120	134		
Middle	14	68		
Total	134	202	11.76	*P*<0.001
Storage practice				
In containers with lid	88	190		
In containers without	46	12		
lid				
Total	134	202	14.73	*P*<0.001

The extent of iodization of salt was determined using the iodometric titration method. It was observed that crystalline salts collected from all retailers had an iodine content <15 ppm, whereas refined salts collected from 30 (90.9%) retailers had an iodine content >30 ppm. About 48.5% of the salt samples collected from retail shops were adequately iodized [Table 3].

**Table 3:** lodometric titration of sample salt at the retailer level

	Crystal (%)	Refined (%)
Titration		
< 1 5 ppm	33(100)	1 (3.0)
15–30 ppm	0(0)	2(6.1)
> 30 ppm	0(0)	30 (90.9)
Total	33(100)	33(100)

From among 33 retailers, 22 (66.7%) were keeping the crystalline salt in uncovered gunny bags/plastic containers and 11 (33.3%) retailers were keeping the crystalline salt in covered gunny bags/plastic containers. All the retailers were keeping refined salt in polythene packets as packaged before at the production level. Out of 33 shopkeepers, 23 (69.7%) had stored the crystalline salt inside the shop and 10 (30.3%) had stored the crystalline salt outside the shop. All the retailers stored refined salt inside the shop.

## Discussion

In the present study, 336 households and 33 retail shops from 11 urban slum areas of Cuttack were studied. This study revealed that more than 60% of the households were using salt samples containing 15 ppm or more of iodine, which is a positive achievement of the USI program but further strengthening of USI efforts is required so that more than 90% of the households can consume adequately iodized salt thus fulfilling the criterion for tracking progress towards eliminating IDD.(1,5)

In a cross-sectional, community-based study conducted in Orissa (State Govt. of Orissa in collaboration with NIN, AIIMS, ICCIDD, UNICEF), it was observed that the proportion of households consuming adequately iodized salt (> 15 ppm) was 45% and approximately 47.7% of the salt samples collected from retail shops were adequately iodized.(6) In a cross-sectional, community-based study conducted in Kerala, it was found that 48.9% of the households were consuming adequately iodized salt and the proportion of retail shops selling adequately iodized salt was 61%.(7) In another cross-sectional, community-based study conducted in Bihar, 40.1% of the households were found to be consuming adequately iodized salt.(8)

Iodine deficiency was significantly marked in sample salts collected from katcha houses as compared with salts from pucca houses, which might be attributed to high moisture content in katcha houses. Again, the iodine deficiency in the sample salts was significantly marked in households with low financial status, which indicates that people with low income preferred to buy the unbranded, crystalline loose salt as it is cheaper than the branded, packeted salt.

In all retail shops, crystalline salt was sold along with different varieties of refined salts. The crystalline salts collected from all retailers were found to have an iodine content <15 ppm i.e., inadequately iodized. Again 51.5% of the salt samples collected from the retailers were found to be inadequately iodized, which meant people living in the slums were likely to consume this salt because of its lower price. Out of 33 retailers, 22 (66.7%) were keeping the crystalline salt in uncovered gunny bags/plastic containers and 10 (30.3%) were storing the crystalline salt outside the shop, which might cause a loss of iodine due to exposure to sunlight and moisture.

## Recommendations

The following points are recommendations based on the findings of this study:

The crystalline salts collected from all retailers were inadequately iodized and more than one third of the households were consuming crystalline salt. Therefore, it becomes vital to adequately iodize all crystalline salts. The people living in the slums should be properly educated regarding storage practices of edible salt.

There should be an appropriate mechanism for providing adequately iodized salt to households with low percapita monthly income at a price they can afford.
